# Intelligent Segmentation Medical Assistance System for MRI Images of Osteosarcoma in Developing Countries

**DOI:** 10.1155/2022/7703583

**Published:** 2022-01-19

**Authors:** Jia Wu, Shun Yang, Fangfang Gou, Zhixun Zhou, Peng Xie, Nuo Xu, Zhehao Dai

**Affiliations:** ^1^School of Computer Science and Engineering, Central South University, Chang sha 410083, China; ^2^Department of Spine Surgery, The Second Xiangya Hospital, Central South University, Changsha 410011, China

## Abstract

Osteosarcoma is the most common primary malignant bone tumor in children and adolescents. It has a high degree of malignancy and a poor prognosis in developing countries. The doctor manually explained that magnetic resonance imaging (MRI) suffers from subjectivity and fatigue limitations. In addition, the structure, shape, and position of osteosarcoma are complicated, and there is a lot of noise in MRI images. Directly inputting the original data set into the automatic segmentation system will bring noise and cause the model's segmentation accuracy to decrease. Therefore, this paper proposes an osteosarcoma MRI image segmentation system based on a deep convolution neural network, which solves the overfitting problem caused by noisy data and improves the generalization performance of the model. Firstly, we use Mean Teacher to optimize the data set. The noise data is put into the second round of training of the model to improve the robustness of the model. Then, we segment the image using a deep separable U-shaped network (SepUNet) and conditional random field (CRF). SepUnet can segment lesion regions of different sizes at multiple scales; CRF further optimizes the boundary. Finally, this article calculates the area of the tumor area, which provides a more intuitive reference for assisting doctors in diagnosis. More than 80000 MRI images of osteosarcoma from three hospitals in China were tested. The results show that the proposed method guarantees the balance of speed, accuracy, and cost under the premise of improving accuracy.

## 1. Introduction

Osteosarcoma is the most common primary bone tumor [1], mostly in children and adolescents. The incidence rate of osteosarcoma in the world is the highest in all primary malignant bone tumors (44%). Especially in developing countries, due to the limitation of medical level, the death toll accounts for a higher proportion than that in developed countries. In China, though the overall incidence rate is not high, the incidence of [2] is more than 2000. Most patients showed the characteristics of a high degree of malignancy and poor prognosis. The 5-year survival rate of patients with advanced osteosarcoma is only about 20% [3]. If it can be detected early and treated in time, it can greatly improve the survival rate of patients and reduce the probability of amputation [4]. Because magnetic resonance imaging (MRI) has good soft-tissue resolution and very high contrast resolution and its multiparameter and multiplane slicing capability can clearly show the location and extent of the lesion, the damage to the human body during the detection process is minimal. Therefore, MRI is a common imaging technique used by doctors to diagnose and evaluate osteosarcoma.

Most developing countries have encountered obstacles in the diagnosis, treatment, and prognosis of osteosarcoma due to the general imperfect medical system. The developing countries are economically backward, and medical resources are in short supply [5–8]. The high-priced magnetic resonance imaging equipment and the lack of professional talents make the early diagnosis of osteosarcoma very difficult [9–11]. In addition, the diagnosis of osteosarcoma at this stage relies on manual identification by doctors [12–14]. Each patient will produce 600-700 MRI images at one diagnosis [12]. In a large amount of data, often less than 20 images are valid. A large amount of redundant data brings a huge workload to doctors, leading to inefficient diagnosis [13]. Worst of all, the location, structure, size, and shape of different osteosarcomas vary from person to person, and their distribution density is uneven [14]. The tumor tissue is often indistinguishable from the surrounding normal tissue. Especially in imaging, the images of different osteosarcomas under the same imaging method are also different [15–17]. Sometimes it is difficult to distinguish between normal tissues and diseased areas with the naked eye. Image interpretation is limited by the subjectivity of doctors, doctors' perceptions of huge differences and fatigue, and the rate of misdiagnosis by inexperienced doctors has risen [18].

In recent years, medical image processing technology has to some extent alleviated the difficulties in the diagnosis of osteosarcoma in developing countries [19]. Accurately measuring the area of the tumor area through computer technology can assist doctors in qualitative and even quantitative analysis of lesions and other areas of interest, thereby greatly improving the accuracy and reliability of medical diagnosis [20]. The existing medical image processing technology can detect the position and edge of the tumor to a certain extent. However, the position, shape, and scale of the tumor area vary greatly, and the different degrees of brightness between the images lead to poor interpretation of the model [21]. Therefore, the effect of the existing technology on image segmentation of osteosarcoma has not reached expectations [22].

More and more researches use machine learning methods to optimize the segmentation effect. Many methods use many selected features to learn the mapping relationship from the feature space to the training label, thereby improving the accuracy of tumor segmentation [22]. However, these features need to be extracted manually, the implicit features of the image cannot be considered, and training a classifier with many features is a time-consuming and costly task [23, 24]. At the same time, the structure, shape, and location of osteosarcoma are complex, and there is a lot of noise in MRI images, which will cause the model to overfit [25]. Many studies have used complex structures and deeper levels to optimize their fitting capabilities so that the model has stronger generalization. Although this method can improve the accuracy of the model to a certain extent, the improvement effect of such methods in segmentation accuracy is often small. Moreover, an overly complex structure will make the training of the model slow and inefficient.

Based on the above analysis, this paper proposes an osteosarcoma-assisted segmentation method (OSDCN) based on a deep convolutional neural network. First, we expanded the original data set to reduce the degree of overfitting and enhance the generalization performance of the model. At the same time, we use the Mean Teacher algorithm to optimize the data set to reduce the influence of the difference between the brightness of MRI images on the model training. Further, we use the binarization algorithm to screen the effective area in the MRI image, reducing the waste of resources and computational cost. In terms of model design, taking into account the uneven image of osteosarcoma and the complicated tumor shape, we used a depth-separable U-shaped network (SepUNet) to segment tumors of different sizes at multiple scales according to features of different depths. Moreover, we added the conditional random field on this basis to further optimize the segmentation results and solve the problem that the tumor is more blurred than the boundary. Finally, to provide doctors with more intuitive analysis results, we calculated the tumor area of the three sections of the human body in the patient's MRI image. The OSDCN method plays an extremely important role in the diagnosis, treatment, and prognosis of osteosarcoma.

The detailed contributions of this research are as follows:

1. This article optimizes and preprocesses the original data set. The Mean Teacher optimization algorithm alleviates the influence of noise tags on model training and supplements the valuable knowledge of high-loss blocks. Standardized preprocessing reduces the influence of image sensitivity caused by external factors on the model's segmentation of tumor regions. At the same time, ineffective areas are shielded to reduce waste of resources and training costs
2. This article integrates the deep separable U-shaped network and conditional random field as the image segmentation model, which can not only accurately lock the tumor regions of different sizes in the MRI image but also further locate the tumor boundary, improving the accuracy of segmentation and model training.
3. In the calculation method of tumor area, this paper uses particle filter technology to fit the boundary curve, which improves the accuracy of boundary positioning. At the same time, the complex Newton-Cotes algorithm is applied to area calculation, which avoids the rounding error of high-order interpolation and further subdivides the area interval to improve the accuracy of area calculation
4. We used more than 80,000 samples collected from the Second Xiangya Hospital of Central South University for experimental analysis. The results show that our proposed osteosarcoma segmentation method is superior to other methods. This method plays a significant role in the diagnosis, treatment, and prognosis of osteosarcoma. Doctors use the result of diagnosis as an auxiliary basis for diagnosis and treatment, which can reduce workload and time without affecting the accuracy of diagnosis

The content of the other chapters of this article is organized as follows: In Section 2, we give a brief introduction to the relevant work in the research process. In Section 3, we design a segmentation method for osteosarcoma (OSDCN), then describe and analyze each submodule. In Section 4, we report the process and results of the experiment and conduct evaluation and analysis. In the last Section 5, we summarized the full text and looked forward to future work.

## 2. Related Works

There are already many artificial intelligence decision systems and image processing methods used to assist in the diagnosis of diseases. In the diagnosis of osteosarcoma, processing images through computer technology to analyze the health of patients has become a research hotspot. Some mainstream algorithms are introduced below.

Osteosarcoma cells have multiple morphologies, and pathologists disagree on the classification of osteosarcoma (surviving tumor, necrotic tumor, nontumor). Chang et al. [26] proposed a deep model with Siamese network (DS-Net) for automatic classification in Hematoxylin and Eosin (H&E) stained histological images of osteosarcoma, which in turn helps pathologists to improve diagnostic accuracy. To further achieve zero-error classification, Zhan et al. [27] proposed a novel convolutional neural network architecture consisting of multiple CNNs in series, called C-Net. The architecture is divided into outer, middle, and inner parts. Among them, the outer and middle parts of the architecture contain six CNNs as feature extractors to feed the internal network to achieve the classification of malignant and benign tumor images. Similarly, Anisuzzaman et al. [28] provided a solution for automatic detection of osteosarcoma through transfer learning techniques using a CNN pretrained on a public data set of histological images of osteosarcoma. This allows patients with osteosarcoma to be treated at an early stage and avoid more extensive metastases in other bones and soft tissues.

However, the borderline cases of Ewing's sarcoma and osteosarcoma remain a challenging task for medical diagnosis. A Huang et al. [29] used diffusion-weighted imaging (DWI) to achieve precise delineation of Ewing's sarcoma and osteosarcoma by evaluating the apparent diffusion coefficient (ADC) values. And in the past decade of applying deep learning to medical images, convolutional object detection (COD) has also become a successful method for cancer analysis. D'Acunto et al. [30] used a method based on convolutional object detection for differentiating osteosarcoma cells from osteoblasts (MSC). This method shows an accuracy close to 1 on the available data set, which is conducive to effective analysis of single cells, while avoiding traditional biochemical methods that are time-consuming and may require a large number of cells.

To evaluate the grade of osteosarcoma in patients, Gou and Wu [20] proposed a sequential recurrent convolutional neural network (RCNN) model combining convolutional neural network and bidirectional gated recurrent unit (GRU), but the model is prone to an overfitting problem. Similarly, to estimate the case-level necrosis rate, Ho et al. [31] proposed Deep Interactive Learning (DIaL), an effective labeling method for training CNNs. Treatment response, measured as the ratio of necrotic tumor area to the whole tumor area, is a known prognostic factor for overall survival. The DIaL method is mainly used for multiclass tissue segmentation of histopathological images and treatment reflective assessment of osteosarcoma. The main idea is to calculate the number of pixels predicted as live and necrotic tumors by the segmentation model and compare it with the rate in the pathology report, then estimate the case level necrosis rate to provide a more accurate and effective treatment plan for patients. This method can assist doctors in effectively improving the survival rate of patients.

There are also many methods in the literature that use image processing and computer techniques to predict the response to osteosarcoma treatment and its corresponding indicators. To predict chemotherapy response in osteosarcoma and to determine treatment plans for osteosarcoma patients as early as possible, Jeong et al. [32] used baseline 18-FDG positron emission tomography (PET) combined with a machine learning approach for texture feature prediction of the scanned images and then assessed the ability to respond to chemotherapy by the area under the operating characteristic curve (AUC). Im et al. [33] used Otsu (MO-PET), gradient-based method (PETedge), relative threshold method, and background threshold method to segment artificial lesions in the phantom. The metabolic tumor volumes (MTV) using MO-PET and PETedge were named MTV (MO-PET) and MTV (PETedge), respectively. MTV (MO-PET) shows excellent reproducibility and can predict EFS in patients with osteosarcoma.

In addition, Kayal et al. [25] used diffusion-weighted imaging (DWI) to segment osteosarcoma, which plays a crucial role in the diagnosis and prognosis of osteosarcoma. Alge et al. [34] used X-rays to detect the size and location of tumors and combined images and RNA-seq data to distinguish osteosarcoma from benign tumors. Shuai et al. [35] proposed a network architecture W-net++ based on two cascaded U-Nets and dense jump connections to realize automatic segmentation of osteosarcoma lesions in CT images. Huang et al. [36] proposed a fully automated MRI segmentation and recognition method for osteosarcoma. This method mainly uses conditional random fields to identify tumors with various shapes and irregular structures and has achieved good results.

The above analysis shows that artificial intelligence technology has played an increasingly important role in the diagnosis and prognosis of diseases. However, MRI images of osteosarcoma are susceptible to noise, and the edge features are still difficult to maintain well. The segmentation accuracy needs to be further improved. To make up for the lack of segmentation accuracy, we propose an osteosarcoma MRI image segmentation method based on a deep convolutional neural network. This method improves the accuracy of osteosarcoma detection through strategies such as data set optimization, preprocessing, model segmentation, and edge optimization.

## 3. Methods

Due to the serious imbalance of the doctor-patient ratio in developing countries, it is difficult for doctors to provide one-to-one services to patients. At the same time, the diagnosis and treatment cycle of osteosarcoma is long, and the cost is high. Many families cannot afford the high medical expenses, and some people even choose to stop treatment. Most developing countries face economic and technical challenges in the diagnosis and treatment of osteosarcoma. In particular, the MRI images of osteosarcoma are complex, and the amount of data is large. It is very challenging to rely on doctors for manual screening and detection. With the development of smart medicine, image processing is playing an increasingly important role in the diagnosis, treatment, and prognosis of diseases. The system decision-making results can be used as an auxiliary basis for doctors' clinical diagnosis, reduce the doctor's ineffective workload, improve the doctor's work efficiency, and provide more quality services to patients. While improving the efficiency and accuracy of model segmentation, our method should have broader practicability and hardware requirements. In addition, we hope that the system can provide doctors with more intuitive analysis results. Based on this, this paper proposes an osteosarcoma segmentation method (OSDCN) based on a deep convolutional neural network, which is mainly used to assist doctors in identifying MRI images of osteosarcoma, to diagnose osteosarcoma more efficiently and accurately. It can not only accurately identify the MRI image of osteosarcoma and delineate the tumor area in the picture but also calculate the area of the tumor area to provide doctors with more intuitive results. The overall design of this article is shown in Figure 1.

This paper is divided into two sections: Section 3.1 is the segmentation of osteosarcoma MRI images, and Section 3.2 is the calculation of the tumor region area in the model segmentation results. In Section 3.1, we input the MRI images of osteosarcoma patients into the segmentation network, through which we can obtain the location and range of suspicious tumors. It has good effects for subsequent doctors to determine the degree of soft tissue invasion and determine the therapeutic effect.

After processing the MRI images of osteosarcoma in Section 3.1, in Section 3.2, the boundary curve was fitted using the particle filter algorithm, and then, the tumor region area was calculated using the multiplexing Newton-Cotes algorithm.

We list some of the symbols used in this paper in Table 1.

### 3.1. Osteosarcoma Image Segmentation

The overall design of segmentation of osteosarcoma is shown in Figure 1, which is mainly divided into three major structures: optimized data set, preprocessing, image analysis, and segmentation.

To further improve the accuracy of detection, we have set up three strategies:

1. *Data Set Optimization*. Using the Mean-Teacher model to divide the data set into Useful-Slices (US) and Normal-Slices (NS) and input them into the network for training
2. *Pretreatment*. We further preprocess the filtered MRI image to reduce the effective segmentation area and reduce the waste of resources caused by the invalid area
3. *Image Analysis and Segmentation*. The segmentation model in this paper includes two parts: a deeply separable U -shaped model (SepUNet) and a conditional random field (CRF). When training the model, the four perspectives of the same MRI image are input to the network to reduce the false detection rate of the algorithm

#### 3.1.1. Data Set Optimization

The initial data set has a large amount of data. We observe the data set and find that not all slices in a series are good for training, and there are some images with very small tumor regions (some even do not contain tumor regions). Although these samples contain noisy labels, they can also contribute to the model. Therefore, it is not feasible to discard this part of the data directly. However, since deep neural networks can memorize all training samples, directly using these slices may lead to a sharp decline in model performance. Therefore, we need a way to divide useful slices (US) and difficult slices (NS) and can continuously process newly added slice sets.

To solve the first problem, we set ResNet-7 to divide the data set, as shown in Figure 2. ResNet-7 is composed of 6 layers of residual modules plus a layer of fully connected modules. The residual module uses the residual idea to avoid the disappearance of gradients. The final fully connected layer is responsible for classification. A 3 × 3 maximum pooling layer is set between each layer to reduce the size of the feature map.

In addition, to further improve the accuracy and robustness of the division and to better adapt to the newly added slice set, we use the Mean-Teacher semisupervised algorithm. The overall architecture of dividing the network includes two parts: student model and teacher model; that is, there are two ResNet-7 models. Their parameter groups are *θ*_*s*_ and *θ*_*t*_, respectively. The original data set is randomly divided into *X*_1_ (70%) and *X*_2_ (30%), which *X*_1_ have label *Y*_1_, *X*_2_ no labels. The training process of the algorithm is as follows:

1. Input *X*_1_ and *X*_2_input into the student model, output the predicted probability *P*_*s*1_, *P*_*s*2_; input *X*_2_ into the teacher model, output the predicted probability *P*_*t*2_
2. Calculate loss values *l*_1_ according to *P*_*s*1_, *P*_*t*1_, and the loss function *L*_1_. According to the literature [37], the calculation formula of the loss value is

(1) $$\begin{array}{c} L_{1}=-\frac{1}{N}\overset{N}{\underset{i=0}{\sum }}y_{i}∙\log\left(p_{i}\right)+\left(1-y_{i}\right)∙\log\left(1-p_{i}\right),y_{i}\epsilon Y_{1},p_{i}\epsilon P_{s1}. \end{array}$$

(3) Calculate loss values *l*_2_ according to *P*_*s*2_, *P*_*t*2_, and the loss function *L*_2_
(4) The loss value of the student model is *l* = *l*_1_ + *l*_2_, with this gradient descent and updated the parameter to  *θ*_*s*_′. The teacher model [38] updates the parameters *θ*_*t*_′ by moving average (as shown in formula (2)).

(2) $$\begin{array}{c} \theta_{t}^{\prime }=\alpha \theta_{t}+\left(1-\alpha \right)\theta_{s}^{\prime }. \end{array}$$

Among them, because of the existence of the label *X*_1_, the loss function *L*_1_ is a cross-entropy loss function, as shown in formula (1). And *X*_2_ has no label, so *L*_2_ needs to use the Kullbac-Leibler (KL) Divergence relative entropy loss function [39]. Relative entropy is often used to describe the degree of overlap of two distributions. If it completely overlaps, its value is 0, and if it does not overlap, its value is 1. The KL formula is shown below:

(3) $$\begin{array}{c} \text{KL}\left(\left.Q\right\|P\right)=\sum p\left(x\right)∙\log\frac{p\left(x\right)}{q\left(x\right)}. \end{array}$$

However, the KL function has always had a problem of asymmetry. We hope that the prediction distributions of the teacher model and the student model are as consistent as possible, but it is impossible to judge whose prediction is more accurate. Therefore, we quoted the Jenson-Shannon (JS) algorithm [23] to compensate for the asymmetry problem, which is *L*_2_ calculated as:

(4) $$\begin{array}{c} L_{2}=\frac{1}{2}KL\left(\left.P_{s2}\right\|P_{t2}\right)+\frac{1}{2}\text{KL}\left(\left.P_{t2}\right\|P_{s2}\right). \end{array}$$

Finally, the original data set is divided into two parts, the proportion of US is 41.7%, and the proportion of NS is 58.3%, and they are successively input to the segmentation network. The purpose of this is to let the deep network learn simple samples first and get a lower loss value. Research shows that an easy sample is more beneficial to network training.

#### 3.1.2. Pretreatment

In an MRI image of osteosarcoma, we found that the effective area containing bones and flesh only occupies a part of the image, and the other part of the area does not contain any effective information, which is undoubtedly a waste of network segmentation for subsequent images. In addition, it may also interfere with the final result because the gray value of the tumor area after T1-weighted is similar. Therefore, we chose to block this type of area.

As shield invalid region in Figure 3 shown, it is divided into the following three steps:

1. Binarization

In MRI images, the gray value of the body structure is often brighter, while the background pixels that do not contain useful information are often darker. To better distinguish them at the beginning of the experiment, we used a binarization algorithm [40] to classify the pixels according to their gray values. The threshold formula for the algorithm is as follows:

(5) $$\begin{array}{c} T=\text{argmax}\left(\overset{255}{\underset{i=0}{\sum }}\left(\rho_{0}*n_{\text{val}<g}*{\left(\mu -\mu_{\text{val}<g}\right)}^{2}+\rho_{1}*n_{\text{val}\geq g}*{\left(\mu -\mu_{\text{val}\geq g}\right)}^{2}\right)\right), \end{array}$$

where *i* represents the gray value, *ρ*_0_ and *ρ*_1_ are both hyperparameters, *ρ*_0_= 0.67 and *ρ*_1_= 0.33. *n*_val<*g*_ represents the number of pixels with a gray value less than *g*. *μ*_val≥*g*_ representing all gradation values equal to or greater than  *g* the average gray value of the pixel.

When we obtain the threshold of the original image, we set the pixels in the original image that are greater than or equal to the *T* value as bright spots and the pixels less than the *T* value as dark spots.

(2) Deleting isolated bright spots and making up the hollow area

After the binarization of the image, there are sporadic small bright spots in some areas, which increases the difficulty of preprocessing (these small bright spots do not exist in the osteosarcoma area), so the closed operation is used to remove them.

In addition, we found that some dark spots close to the bright spot may also belong to the tumor area, so we started the calculation to set this part of the pixel as the bright spot.

(3) Determining the credible area

The osteosarcoma data set roughly has three types of slices: cross-section, coronal plane, and sagittal plane. Their gray value distribution, lesion area, and shape are all different, so to meet the premise that the lesion area must be included, we set MAX − *X*/MIN − *X* as the bright spot coordinate The maximum/minimum value in the horizontal direction, MAX − *Y*/MIN − *Y* is the maximum/minimum value in the vertical direction, and finally, [MIN − *X* : MAX − *X*, MIN − *Y* : MAX − *Y*] is set as the credible area, and there is no tumor in the noncredible area.

#### 3.1.3. Image Analysis and Segmentation

Osteosarcoma tumor network model for segmentation is based on a multilayer deep separable full convolution neural U Network (SepUNet) [36], as in Figure 4. In the neural network, the deeper the feature receptive field, the larger the area with the larger size. SepUNet can segment tumor regions of different sizes at multiple scales based on features of different depths. This is why it can accurately segment objects. SepUNet is mainly composed of the following three structures:

1. *Encoder*. It is the main structure for extracting image features, with a total of 4 layers. There is a 3 × 3 maximum pooling layer between each layer, which can reduce the size of the feature map to extract features more deeply. Each layer is composed of a DoubleConv and a SeparableBlock. The SeparableBlock is mainly composed of depth separable convolution. Compared with ordinary convolution, it can have higher depth and accuracy under the premise of the same amount of parameters
2. *Decoder*. It is mainly responsible for multiscale features, and there are 4 layers in total. The feature map size between each layer will be enlarged by 2 times through interpolation. Each layer consists of a DoubleConv, which is used to process the combined context characteristics
3. *Skip-Connection*. It is responsible for combining the shallow features of the same-level Encoder with the deep features of the Decoder. This method of combining contextual features is the key to a good segmentation effect of the UNet network

For the artificial intelligence model, the rotated image is a brand new image. The network will focus on different features for segmentation. Therefore, to make the model segmentation result more accurate and robust, we put a picture into the network segmentation after being rotated by 90°, 180°, and 270°. The final segmentation probability is the probability-weighted average of the four images. The calculation formula is as follows shown:

(6) $$\begin{array}{c} \text{Result}=\overset{h}{\underset{i=0}{\sum }}\overset{w}{\underset{j=0}{\sum }}\left(\alpha_{0}p_{0,ij}+\alpha_{1}p_{1,ij}+\alpha_{2}p_{2,ij}+\alpha_{3}p_{3,ij}\right),\overset{3}{\underset{k=0}{\sum }}\alpha_{k}=1. \end{array}$$

After testing, the weight parameter *a*_0_ = 0.4, *a*_1_ = *a*_2_ = *a*_3_ = 0.2. Segmenting fuzzy boundaries has always been a big problem in image segmentation tasks. By observing the MRI image of osteosarcoma, we can find that the edema area, muscle area, and tumor area in the image are very close, and the gray value at the junction is also similar. Even experienced doctors may admit mistakes, which will affect the judgment of the disease. To further reduce the false detection rate, we use a CRF (CRF) to further optimize the boundary of the results after network segmentation.

For the probability map output by the neural network *U*, we can use the following formula (7) to describe the predicted value of each pixel [36]. *X* = {*x*_1_, *x*_2_, ⋯, *x*_*n*_} represents the feature point of each pixel on the probability map, and *Y* = {*y*_1_, *y*_2_, *y*_3_, ⋯, *y*_*n*_} represents the label predicted by each point based on its texture, gray value, and other attributes, and the probability of the surrounding points.

(7) $$\begin{array}{c} P\left(y\;|\;x\right)=\frac{1}{Z\left(x\right)}\exp\left(\underset{i\epsilon U}{\sum }\underset{j\in U\left(x_{i}\right)}{\sum }T_{i,j}\left(y_{j},y_{i},x_{i},i\right)+\underset{i\epsilon U}{\sum }S_{i}\left(y_{i},x_{i}\right)\right). \end{array}$$

Among them, *U*(*x*_*i*_) represents the points around *x*_*i*_, *T*_*i*,*j*_ is the function of the feature transfer between the *i*-th point and the surrounding points, *S*_*i*_ is the state feature function about the *i*-th point, and *Z*(*x*) is the normalized function. According to the literature [36], its calculation is as follows:

(8) $$\begin{array}{c} Z\left(x\right)=\underset{y\epsilon Y}{\sum }P\left(y\;|\;x\right). \end{array}$$

#### 3.1.4. Loss Function

Segmentation of osteosarcoma is a two-class segmentation task. The log loss function is a classic loss function. The log loss function (BCE) formula [41] is shown below, where the probability of each pixel belonging to the osteosarcoma region is *p*_*i*,*j*_; the label is *y*_*i*,*j*_.

(9) $$\begin{array}{c} L_{\text{BCE}}=\frac{1}{h*w}\overset{h}{\underset{i=0}{\sum }}\overset{w}{\underset{j=0}{\sum }}-\left(y_{i,j}*\log\left(p_{i,j}\right)+\left(1-y_{i,j}\right)*\log\left(1-p_{i,j}\right)\right). \end{array}$$

Osteosarcoma segmentation is a small target segmentation task. There is often only one target area in an image, and the corresponding area ratio is not large. If only the logarithmic loss function is used, then the loss gradient pays more attention to the category with a larger area, because this function has the same degree of attention to each pixel, which will eventually make the model lose its predictive ability. So we also need to use the Dice loss function [41], which calculates the loss value for each category and can solve the problem of sample imbalance. The Dice loss function is as follows:

(10) $$\begin{array}{c} L_{\text{Dice}}=1.0-\frac{2.0*\left(\text{GT}\cap P_{\text{os}}\right)}{\left|\text{GT}\right|+\left|P_{\text{os}}\right|}. \end{array}$$

Among them, GT represents the real osteosarcoma region, *P*_os_ represents the predicted osteosarcoma region, and ∣*X*| represents the area of the *X* region. However, if we only use the Dice loss function because of the small area, the prediction bias at several pixels in osteosarcoma may cause unstable gradient changes.

After weighing the stability and accuracy of training, we choose to use the two-loss functions together to alleviate the problems caused by the other loss function. Therefore, the total loss function formula for training is as follows:

(11) $$\begin{array}{c} L=\alpha_{1}L_{\text{BCE}}+\alpha_{2}L_{\text{Dice}},\alpha_{1}+\alpha_{2}=1. \end{array}$$

After experiments, we set the weight parameters *α*_1_ = 0.5 and *α*_2_ = 0.5.

### 3.2. Calculation of Tumor Area

In the imaging of osteosarcoma, MRI can clearly understand the extent of tumor invasion. To provide doctors with more references, we calculated the area of the tumor area of the osteosarcoma segmentation result in the MRI image, as shown in Figure 1.

#### 3.2.1. Introduction to Complex Newton-Cotes

The complex of Newton-Cotes algorithm [42] to calculate the area, both to avoid higher-order interpolation rounding error, in turn further subdivided area range, to improve the area calculation accuracy. Therefore, we use the complex Newton-costs algorithm to calculate the area of the tumor area.

The detailed description of the complex Newton-Cotes algorithm is as follows:

1. *Fitting the Unknown Curve*. Input the initial value *u*_0_, *u*_1_, ⋯, *u*_*n*_ of the node and its corresponding function value *f*(*u*_*r*_)(*r* = 0, 1, ⋯, *n*)(*r* = 0, 1, ⋯, *n*), and obtain the unknown curve fitting equation *F*(*x*) by the following interpolation formula

(12) $$\begin{array}{c} L_{n}\left(u\right)=\overset{n}{\underset{r=0}{\sum }}f\left(u_{r}\right)l_{r}^{\prime }\left(u\right). \end{array}$$

Among them, *l*′_*r*_(*u*) is the interpolation basis function [42]:

(13) $$\begin{array}{c} l_{r}^{\prime }\left(u\right)=\overset{n}{\underset{j=0,j\neq r}{\prod }}\frac{u-u_{r}}{u_{r}-u_{j}}. \end{array}$$

(2) *Dividing the Integrand Interval*. Divide the integral interval [*a*, *b*] into ten equal parts, divide points *u*_*r*_ = *a* + *rh*(*r* = 0, 1, 2, 3, ⋯, 10), take a step size of *h* = (*b* − *a*)/10; then divide each subinterval into [*u*_*r*_, *u*_*r*+1_] equal part points; the interior points are recorded as: *u*_*r*+(1/4)_, *u*_*r*+(1/2)_, *u*_*r*+(3/4)_. According to the interpolation type quadrature formula [42], the specific calculation is as follows:

(14) $$\begin{array}{c} I_{n}\left(u\right)=\left(b-a\right)\overset{n}{\underset{r=0}{\sum }}c_{r}^{\left(n\right)}f\left(u_{r}\right). \end{array}$$

Among them, *c*_*r*_^(*n*)^ is the Cotes coefficient.

(3) *Calculate the Tumor Area*. Calculate the area of the tumor area

(15) $$\begin{array}{c} C_{10}=\frac{h}{90}\left[7f\left(a\right)+32\overset{9}{\underset{r=1}{\sum }}f\left(u_{r+\left(1/4\right)}\right)+2\overset{9}{\underset{r=0}{\sum }}f\left(u_{r+\left(1/2\right)}\right)+32\overset{9}{\underset{r=0}{\sum }}f\left(u_{r+\left(3/4\right)}\right)+14\overset{9}{\underset{r=1}{\sum }}f\left(u_{r}\right)+7f\left(b\right)\right]. \end{array}$$

#### 3.2.2. Tumor Area Calculation

We calculate the area of the patient's tumor area, to provide a reference for the doctor's clinical diagnosis. The specific calculation steps are as follows:

**Step 1 .**

Measuring the boundary coordinates of the tested tumor area. Subsequently, the MCMC particle filter algorithm is used to smooth the filtered output and further improve the accuracy. Under conditions precision can be measured at intervals of the boundary region is 1 mm the stippling marked, and identify each tumor region under extreme points left, and right directions, to determine the irregular region located the smallest circumscribed rectangle. As shown in the irregular tumor area in the lower half of Figure 5.

**Step 2 .**

Determining the size of the divided squares. We use a small square of 4 mm × 4 mm to divide the circumscribed rectangular coordinate plane into some small squares of equal size, as shown in the small squares divided in the lower half of Figure 5.

**Step 3 .**

Using the improved grid method to calculate the area of the lesion area. Through the above division method, three types of small squares can be obtained: no overlap, partial overlap, and complete overlap with the measured area.

Situation 1. Grids that do not overlap with the measured area will not be considered when calculating the area.

Situation 2. The overlap area of the *M*_1_ squares that completely overlap the measured area is known, and it is recorded as *S*_*c*_ = 16 mm^2^.

Situation 3. For those *M*_2_ squares that partially overlap with the measured area, the area calculation should be performed using the complex Newton-Cotes algorithm. Boundary curve *f*(*x*)  in Figure 5 on the upper part shown, to a side of the square equal intervals segment 10 parts. Then, use the Newton-Cotes formula once in each cell (i.e., subdivide 4 parts again, at this time, the square is equivalent to 40 parts, and the distance between each split node is 0.01 mm). Finally, the size of the overlapping area with the region can be obtained by the compound Newton-Cotes formula, which is recorded as *S*_*i*_. Figure 5 in the upper half, boundary curve  *f*(*x*), and the area enclosed by the axes.

(16) $$\begin{array}{c} S_{\text{os}}=\overset{M_{2}}{\underset{i=0}{\sum }}S_{i}+M_{1}∙S_{c}. \end{array}$$

**Step 4 .**

Finally, summing the overlapping areas of the small squares in the area to get the total area of the irregular osteosarcoma area, which is calculated as follows. The schematic diagram of the segmentation and fitting process is shown in Figure 5.

After training the model using the MRI images of the cross-section, coronal, and sagittal planes of patients with osteosarcoma, we will finally obtain three types of image segmentation results and the tumor area of the three sections of the human body. In the clinical diagnosis of osteosarcoma, the size of the tumor (T), the presence or absence of regional lymph node invasion (N), and the presence or absence of distant metastasis (M) are all the focus of doctors' attention. Our segmentation system can not only accurately classify osteosarcoma, and it can provide the tumor area of different sections of osteosarcoma in MRI images. Doctors use the results of the segmentation and the final lesion area as an auxiliary basis for diagnosing osteosarcoma, which helps to improve the accuracy of diagnosis.

## 4. Results

### 4.1. Data Set

The data in this article is provided by the Ministry of Education Mobile Health Information-China Mobile Joint Laboratory and the Second Xiangya Hospital of Central South University. In addition, we have collected statistics on images and indicators of hospitals in recent years. From osteosarcoma patients, we have compiled more than 80,000 MRI osteosarcoma images and other index data from 204 patients. To make the model segmentation result more accurate and robust, we put a picture into the network segmentation after being rotated by 90°, 180°, and 270° to obtain the final segmentation result. The specific number of patient information items is shown in Table 2. We choose 80% of the data as the training set and 20% of the data as the test set. There are a total of 204 cases, 164 in the training set, and 40 in the test set.

### 4.2. Evaluation Indexes

To evaluate the performance of the model, we use accuracy, precision, recall, F1-score, Intersection of Union (IOU), and Dice Similarity Coefficient (DSC) as the measurement indicators. A confusion matrix composed of true positives (TP), true negatives (TN), false positives (FP), and false negatives (FN) is used to explain the performance of the network. Among them, TP indicates that it is determined to be an osteosarcoma area, which is an osteosarcoma area. FP indicates that it is judged to be a normal area, but it is also a normal area. FP means that it is judged to be a tumor area, but in fact, it is a normal area. FN indicates that it is judged to be a normal area, but in fact, it is a tumor area. The relevant indicators we defined are introduced as follows:

Accuracy (Acc) is the proportion of all samples that are correctly judged. It is defined as follows:

(17) $$\begin{array}{c} \text{Acc}=\frac{\text{TP}+\text{TN}}{\text{TP}+\text{TN}+\text{FP}+\text{FN}}. \end{array}$$

Precision (Pre) indicates the proportion of true positive samples among the judged positive samples. It is defined as follows:

(18) $$\begin{array}{c} \text{Pre}=\frac{\text{TP}}{\text{TP}+\text{FP}}. \end{array}$$

Recall (Re) represents the proportion of correctly predicted positive samples to actual positive samples, and it is defined as follows:

(19) Re=TPTP+FN,F1=2∗Pre∗RePre+Re.

F1-score (F1) is based on Precision and Recall. The higher the value of F1, the better the robustness of the model. Its calculation formula is as follows: IOU represents the similarity between the predicted tumor area and the real tumor area. Dice Similarity Coefficient (DSC) is the similarity of the sample; the range is 0-1. When DSC is 1, the segmentation result is the best. We set *I*_1_ as the judged tumor area and *I*_2_ as the real tumor area. Then, IOU represents the ratio of the intersecting area in the two areas. DSC represents the ratio of twice the area of the intersecting area to the sum of the areas of *I*_1_ and *I*_2_.

(20) $$\begin{array}{c} \text{IOU}=\frac{I_{1}\cap I_{2}}{I_{1}\cup I_{2}},\\ \text{DSC}=\frac{2*\left|I_{1}\cap I_{2}\right|}{\left|I_{1}\right|+\left|I_{2}\right|}. \end{array}$$

In addition, we use Params to represent the number of model parameters, The larger the value, the more storage space the model needs. Floating point operation (FLOP) is used to measure the computational complexity of the model. In the segmentation of MRI images of osteosarcoma, we try to increase the recall rate (Recall) as much as possible to avoid the occurrence of missed diagnosis.

### 4.3. Comparison Algorithm

We used FCN [43], PSPNet [44], MSFCN [45], MSRN [24], Unet [46], FPN [47] algorithms, and our proposed OSDCN for comparative experimental analysis. Here is a brief introduction to these methods:

1. Fully convolutional network (FCN) classifies images at the pixel level and uses skip structures to achieve fine segmentation [43]. It can accept input images of any size and use the deconvolution layer to upsample the feature map of the last convolution layer. This article uses FCN-8s and FCN-16s networks with 8 times upsampling and 16 times upsampling
2. The core of Pyramid Scene Parsing Network (PSPNet) is the pyramid pooling module, which can aggregate the context information of different regions, so as to have a good effect in obtaining global information [44]
3. MSFCN is an automatic tumor segmentation network based on a multisupervised output layer full convolutional network [45]. It uses multiple feature channels in the upsampling part to capture more contextual information, thereby ensuring accurate tumor segmentation
4. Multiscale Residual Network (MSRN) [24] based on the residual block introduces convolution kernels of different sizes, adaptively detects image features of different scales, and obtains the most effective image information at the same time. It makes full use of the characteristics of low-resolution images
5. U-net is a U-shaped structure that uses convolution to encode (used below) and then decode (upsampling) [46]. It includes two parts: feature extraction and upper adoption. Compared with other segmentation models, it is simple and efficient
6. Feature pyramid networks (FPN) use both the high-resolution of low-level features and the high-semantic information of high-level features to achieve prediction effects by fusing these features of different layers [47]. And the prediction is performed separately on each fusion feature layer, which is different from the conventional feature fusion method. The results show that FPN has better performance in small object detection

### 4.4. Training Strategy

Before training the segmentation model, to enhance the robustness of the model and avoid excessive attention to meaningless features, we need to enhance the data set. We expanded the data set by zooming in (reducing) the image, rotating the image, and flipping the image.

The training segmentation neural network has been trained for a total of 300 epochs. During training, we set Adam as the optimizer, the initial learning rate is set to 0.001, when the training reaches 200 epochs, the learning rate is changed to 0.0001, and finally, CosineAnnealingLR is used to dynamically adjust the learning rate in the process.

### 4.5. Evaluation of Segmentation Effect

In our model, we divide the data set into Useful-Slices (US) and Normal-Slices (NS). As illustrated in Figure 6, the right figure is the NS image. The boundary between tumor tissue and normal tissue is not clear enough, and the training process is time-consuming and laborious, so we divide it into the NS data set. The left figure clearly shows the segmentation boundary between different organizations, so it is classified as the US data set.

The comparison of model segmentation effect before and after data set processing is shown in Figure 7. The left column is ground truth, the middle column is the segmentation effect diagram of the model before data optimization, and the right column is the segmentation effect of the optimized model. Before optimization, as the middle column shows, there is an incomplete and inaccurate segmentation. After optimization, as the right column shows, the result is closer to the real label, and the completeness and accuracy of the predicted result are both improved. It can be seen that after the optimization of the data set, the performance of the model is significantly promoted.

Figure 8 shows the effect of segmenting MRI images of osteosarcoma by each model. Columns (B)-(H) are the miniature images in the red boxes in column (A). In the images in columns (B)-(H) of Figure 8, the green curve is the truth ground, the red curve is the model-predicted lesion area curve, and the yellow curve is fitted by the green curve and the red curve. We can intuitively analyze the segmentation performance of the model through the proportion of the yellow curve. According to five osteosarcoma segmentation examples, we can find that OSDCN can better segment osteosarcoma and best fit the segmentation standard.

To evaluate the performance of different methods more clearly, we quantify the segmentation results. We use different evaluation indicators for comparative analysis.  Table 3 compares the performance of different methods on the osteosarcoma data set. According to the data in Table 3, the SepUNet model shows good performance in segmenting osteosarcoma tasks, and the model is higher than other models in evaluation indicators such as DSC, IOU, Recall, and F1-score. The model can segment the results more accurately and robustly. While the accuracy of the model is improved, the number of parameters does not increase too much, which also ensures that doctors can get accurate results while the hospital does not need to be equipped with expensive hardware facilities, such as graphics processing units and memory.

Besides, according to Table 3 and Figure 9, we can get that CRF, image preprocessing, and data set optimization are beneficial to improve the prediction results, and it is proved that optimizing the data set can significantly improve the final result and optimize SepUNet's boundary segmentation. Pr increased by about 0.01%, and F1, IOU, and DSC increased by about 0.005% on average. After Prop optimization, the most important DSC index increased by about 0.020%, and Pr, Re, F1, and IOU increased by 0.001%, 0.006%, 0.007%, and 0.014%, respectively.

Figure 10 shows the comparison between the number of parameters of different model methods and DSC. The results show that the segmentation model of osteosarcoma presented by us has the best accuracy with a 2% higher accuracy than the second place. In addition, in terms of the number of parameters, while increasing the accuracy, our model kept a relatively small number of parameters, only 20.32M, far less than 134.3M of FCN-16s and only slightly higher than 17.26M of UNet, which reduced the difficulty of training.

Figure 11 shows the comparison between the FLOPs of different model methods and DSC. The results show that the SepUNet can significantly improve the accuracy and does not need to increase the calculation cost too much and realizes the accuracy-speed trade-off. The performance of Unet model is slightly weaker than our proposed method. But compared with several other models, its performance is also better. Although the segmentation accuracy of MSFCN and MSRN is also high, these two models require very large computational costs.

The changes in the accuracy of each model are shown in Figure 12. We trained a total of 300 rounds, randomly selected 50 rounds (one round per 6 rounds randomly) for display, comparative analysis. It can be seen that after 100 epochs, the accuracy of each model is stable. In numerical value, SepUnet (ours) is the highest, reaching more than 95% stability. The accuracy ranking is SepUnet (ours) > UNet > FPN > FCN-8 s ≈ FCN-16 s > MSRN > MSFCN. At the same time, we selected several models to compare recall rates. As shown in Figure 13, it can be seen from the figure that around 120 epochs before training, the recall rate of Unet, FPN, and MSFCN models fluctuates greatly. After that, all models except the MSRN model have reached a steady state. The data of the MSRN model will fluctuate to a certain extent during the training process. In general, the recall rate of our proposed method is always the highest. It can better avoid the occurrence of missed diagnoses.

Subsequently, we selected four models in the same way and compared F1-score with our method. As shown in Figure 14, it can be seen from the figure that, although the method we proposed has large fluctuations, its F1 value is always the highest. It shows that our model has better robustness. Compared with the segmentation performance of each model in Table 3, the proposed method has a better effect on the MRI data set of osteosarcoma patients. This method can provide a reference for clinical doctors.

## 5. Conclusion

In this paper, more than 80,000 osteosarcoma MRI images from three hospitals in China are used as data sets to propose an osteosarcoma MRI image segmentation model (OSDCN) based on a deep convolutional neural network. The method includes data set optimization, image preprocessing, model segmentation, edge optimization, and tumor area calculation. We compare this method with the classical segmentation model. The experimental results show that our proposed method can significantly improve the accuracy rate and does not need to increase the calculation cost too much. It achieves a trade-off between accuracy and speed.

In the future, with the development of computer technology, we will introduce other information into the method, such as boundary and texture, to solve the segmentation error caused by the small gray difference between tumor tissue and surrounding tissue, and further improve the segmentation accuracy.

## Figures and Tables

**Figure 1:** Framework diagram of the general plan.

**Figure 2:** (a) The flow chart of the Mean-Teacher data set optimization algorithm. (b) The ResNet-7 structure view, teacher model, and student model structure of Figure 1.

**Figure 3:** Flow chart of slice image preprocessing.

**Figure 4:** Architecture design diagram of osteosarcoma segmentation neural network.

**Figure 5:** Schematic diagram of tumor area calculation.

**Figure 6:** Partition of the data set.

**Figure 7:** Comparison of model segmentation effects before and after data set processing.

**Figure 8:** Comparison of segmentation effects of different methods.

**Figure 9:** The performance of the three models proposed by us in different indicators.

**Figure 10:** Parameters of osteosarcoma model and DSC comparison chart.

**Figure 11:** FLOPs of osteosarcoma model and DSC comparison chart.

**Figure 12:** Accuracy changes of each model.

**Figure 13:** Recall changes of each model.

**Figure 14:** F-score changes of each model.

**Table 1:** Some of the symbols and their definitions in this chapter.

Symbol	Paraphrase
*x*_*i*_	The *i*-th training sample
*y*_*i*_	The *i*-th output samples
*X*_1_, *X*_2_	Original data set
*P*_*s*1_	The output probability when the original data is *X*_1_ input to the student model
*P*_*t*2_	The output probability when the original data is *X*_2_ input to the teacher model
*l*	Loss value
*L*_1_	Cross-entropy loss function
*L*_2_	Relative entropy loss function
*L*	Total loss function
*g*	Grayscale value
*X* = {*x*_1_, *x*_2_, ⋯, *x*_*n*_}	The feature point of each pixel on the probability map
*Y* = {*y*_1_, *y*_2_, ⋯, *y*_*n*_}	Probability prediction label for each point.
*T*	Algorithm threshold
*GT*	Real osteosarcoma area
*P*_os_	Predict the area of osteosarcoma
*S*_os_	The area of the tumor area of osteosarcoma

**Table 2:** The baseline of patient characteristics.

Characteristics	Total *N* = 204	Training set *N* = 164 (80.4%)	Test set *N* = 40 (16.9%)
Age			
<15	48 (23.5%)	38 (23.2%)	10 (25%)
15-25	131 (64.2%)	107 (65.2%)	24 (60.0%)
>25	25 (12.3%)	19 (11.6%)	6 (15.0%)
Sex			
Female	92 (45.1%)	69 (42.1%)	23 (57.5%)
Male	112 (54.9%)	95 (57.9)	17 (42.5%)
Marital status			
Married	32 (15.7%)	19 (11.6%)	13 (32.5%)
Unmarried	172 (84.3%)	145 (88.4%)	27 (67.5%)
SES			
Low SES	78 (38.2%)	66 (40.2%)	12 (30.0%)
High SES	126 (61.8%)	98 (59.8%)	28 (70.0%)
Surgery			
Yes	181 (88.8%)	146 (89.0%)	35 (87.5%)
No	23 (11.2%)	18 (11.0%)	5 (12.5%)
Grade			
Low grade	41 (20.1%)	15 (9.1%)	26 (65%)
High grade	163 (79.9%)	149 (90.9%)	14 (35%)
Location			
Axial	29 (14.2%)	21 (12.8%)	8 (20%)
Extremity	138 (67.7%)	109 (66.5)	29 (72.5%)
Other	37 (18.1%)	34 (20.7%)	3 (7.5%)

**Table 3:** Comparison of performance of different methods in MRI images of patients with osteosarcoma.

Model	Pr	Re	F1	IOU	DSC	Params	FLOPs
FCN-16s	0.922	0.882	0.900	0.824	0.859	134.3M	190.35G
FCN-8s	0.941	0.873	0.901	0.830	0.876	134.3M	190.08G
PSPNet	0.856	0.888	0.872	0.772	0.870	49.07M	101.55G
MSFCN [3]	0.881	0.936	0.906	0.841	0.874	20.38M	1524.34G
MSRN [4]	0.893	0.945	0.918	0.853	0.887	14.27M	1461.23G
FPN	0.914	0.924	0.919	0.852	0.888	88.63M	141.45G
UNet	0.922	0.924	0.923	0.867	0.892	17.26M	160.16G

Our (SepUNet)	0.927	0.932	0.930	0.869	0.896	20.32M	199.26G
Our (SepUNet+CRF)	0.939	0.926	0.932	0.874	0.901	20.32M	200.07G
Our (SepUNet+CRF +Prop)	0.937	0.938	0.937	0.883	0.914	20.32M	200.07G

## Data Availability

“Data Availability” statement data used to support the findings of this study are currently under embargo while the research findings are commercialized. Requests for data, 12 months after publication of this article, will be considered by the corresponding author.

## References

[1] Corre I., Verrecchia F., Crenn V., Redini F., Trichet V. (2020). The osteosarcoma microenvironment: a complex but targetable ecosystem. *Cells*.

[2] Saifuddin A., Sharif B., Gerrand C., Whelan J. (2019). The current status of MRI in the pre-operative assessment of intramedullary conventional appendicular osteosarcoma. *Skeletal Radiology*.

[3] Sadoughi F., Maleki Dana P., Asemi Z., Yousefi B. (2021). DNA damage response and repair in osteosarcoma: defects, regulation and therapeutic implications. *DNA Repair*.

[4] Gao S.-S., Wang Y.-J., Zhang G.-X., Zhang W.-T. (2020). Potential diagnostic value of miRNAs in peripheral blood for osteosarcoma: a meta-analysis. *Journal of Bone Oncology*.

[5] Soliman R. M., Elhaddad A., Oke J. (2021). Temporal trends in childhood cancer survival in Egypt, 2007 to 2017: a large retrospective study of 14 808 children with cancer from the Children’s Cancer Hospital Egypt. *International Journal of Cancer*.

[6] Wu J., Gou F., Tan Y. (2021). A staging auxiliary diagnosis model for nonsmall cell lung cancer based on the intelligent medical system. *Computational and Mathematical Methods in Medicine*.

[7] Wu J., Tan Y., Chen Z., Zhao M. (2018). Decision based on big data research for non-small cell lung cancer in medical artificial system in developing country. *Computer Methods and Programs in Biomedicine*.

[8] Wu J., Zhuang Q., Tan Y. J. C. (2020). Auxiliary medical decision system for prostate cancer based on ensemble method. *Computational and Mathematical Methods in Medicine*.

[9] Cui R., Chen Z., Wu J., Tan Y., Yu G. (2021). A multiprocessing scheme for PET image pre-screening, noise reduction, segmentation and lesion partitioning. *IEEE Journal of Biomedical and Health Informatics*.

[10] Wu J., Guan P., Tan Y. J. I. A. (2019). Diagnosis and data probability decision based on non-small cell lung cancer in medical system. *IEEE Access*.

[11] Wu J., Chang L., Yu G. (2021). Effective data decision-making and transmission system based on mobile health for chronic disease management in the elderly. *IEEE Systems Journal*.

[12] Wu J., Tan Y., Chen Z., Zhao M. (2018). Data decision and drug therapy based on non-small cell lung cancer in a big data medical system in developing countries. *Symmetry*.

[13] Yu G., Chen Z., Wu J., Tan Y. (2021). Medical decision support system for cancer treatment in precision medicine in developing countries. *Expert Systems with Applications*.

[14] Wu J., Chen Z. (2016). Data decision and transmission based on mobile data health records on sensor devices in wireless networks. *Wireless Personal Communications*.

[15] Chen H., Xiong W., Wu J., Zhuang Q., Yu G. J. I. A. (2020). Decision-making model based on ensemble method in auxiliary medical system for non-small cell lung cancer. *IEEE Access*.

[16] Yu G., Chen Z., Wu J., Tan Y. J. K.-B. S. (2021). A diagnostic prediction framework on auxiliary medical system for breast cancer in developing countries. *Knowledge-Based Systems*.

[17] Wu J., Tian X., Tan Y. (2019). Hospital evaluation mechanism based on mobile health for IoT system in social networks. *Computers in Biology and Medicine*.

[18] Nasor M., Obaid W. (2021). Segmentation of osteosarcoma in MRI images by K-means clustering, Chan-Vese segmentation, and iterative Gaussian filtering. *IET Image Processing*.

[19] Georgeanu V., Mamuleanu M. L., Selişteanu D. Convolutional neural networks for automated detection and classification of bone tumors in magnetic resonance imaging.

[20] Gou F., Wu J. (2022). Triad link prediction method based on the evolutionary analysis with IoT in opportunistic social networks. *Computer Communications*.

[21] Arunachalam H. B., Mishra R., Daescu O. (2019). Viable and necrotic tumor assessment from whole slide images of osteosarcoma using machine-learning and deep-learning models. *PLoS One*.

[22] Luo Z., Chen W., Shen X. (2020). CT and MRI features of calvarium and skull base osteosarcoma (CSBO). *The British Journal of Radiology*.

[23] Chen H., Liu J., Cheng Z. (2020). Development and external validation of an MRI-based radiomics nomogram for pretreatment prediction for early relapse in osteosarcoma: a retrospective multicenter study. *European Journal of Radiology*.

[24] Zhang R., Huang L., Xia W., Zhang B., Qiu B., Gao X. (2018). Multiple supervised residual network for osteosarcoma segmentation in CT images. *Computerized Medical Imaging and Graphics*.

[25] Baidya Kayal E., Kandasamy D., Sharma R., Bakhshi S., Mehndiratta A. J. S. (2020). Segmentation of osteosarcoma tumor using diffusion weighted MRI: a comparative study using nine segmentation algorithms. *Signal, Image and Video Processing*.

[26] Chang L., Wu J., Moustafa N., Bashir A. K., Yu K. (2021). AI-driven synthetic biology for non-small cell lung cancer drug effectiveness-cost analysis in intelligent assisted medical systems. *IEEE Journal of Biomedical and Health Informatics*.

[27] Zhan X., Long H., Gou F., Duan X., Kong G., Wu J. (2021). A convolutional neural network-based intelligent medical system with sensors for assistive diagnosis and decision-making in non-small cell lung cancer. *Sensors*.

[28] Anisuzzaman D., Barzekar H., Tong L., Luo J., Yu Z. (2021). A deep learning study on osteosarcoma detection from histological images. *Biomedical Signal Processing and Control*.

[29] Huang Z., Li X., Wu J. (2021). An effective data transmission scheme based on IoT system in opportunistic social networks. *International Journal of Communication Systems.*.

[30] D’Acunto M., Martinelli M., Moroni D. (2019). From human mesenchymal stromal cells to osteosarcoma cells classification by deep learning. *Journal of Intelligent & Fuzzy Systems*.

[31] Ho D. J., Agaram N. P., Schüffler P. J. Deep interactive learning: an efficient labeling approach for deep learning-based osteosarcoma treatment response assessment.

[32] Jeong S. Y., Kim W., Byun B. H. (2019). Prediction of chemotherapy response of osteosarcoma using baseline 18F-FDG textural features machine learning approaches with PCA. *Contrast Media & Molecular Imaging*.

[33] Im H. J., Solaiyappan M., Lee I. (2018). Multi-level Otsu method to define metabolic tumor volume in positron emission tomography. *American Journal of Nuclear Medicine and Molecular Imaging*.

[34] Alge O., Lu L., Li Z., Hua Y., Gryak J., Najarian K. Automated classification of osteosarcoma and benign tumors using RNA-seq and plain X-ray.

[35] Shuai L., Gao X., Wang J. Wnet++: a nested W-shaped network with multiscale input and adaptive deep supervision for osteosarcoma segmentation.

[36] Huang W.-B., Wen D., Yan Y., Yuan M., Wang K. Multi-target osteosarcoma MRI recognition with texture context features based on CRF.

[37] Uittenbogaard R., Sebastian C., Vijverberg J., Boom B., Gavrila D. M. Privacy protection in street-view panoramas using depth and multi-view imagery.

[38] Zhou G., Fan Y., Cui R., Bian W., Zhu X., Gai K. Rocket launching: a universal and efficient framework for training well-performing light net.

[39] Ponti M., Kittler J., Riva M., de Campos T., Zor C. (2017). A decision cognizant Kullback-Leibler divergence. *Pattern Recognition*.

[40] Ju Z., Wang C., He X. An improved license plate characters binarization algorithm based on sub-pixel.

[41] Abdeltawab H., Khalifa F., Taher F. Automatic segmentation and functional assessment of the left ventricle using U-net fully convolutional network.

[42] Chen Y. (2021). Study on weighted-based discrete noniterative algorithms for computing the centroids of general type-2 fuzzy sets. *International Journal of Fuzzy Systems*.

[43] Long J., Shelhamer E., Darrell T. Fully convolutional networks for semantic segmentation.

[44] Zhao H., Shi J., Qi X., Wang X., Jia J. Pyramid scene parsing network.

[45] Huang L., Xia W., Zhang B., Qiu B., Gao X. (2017). MSFCN-multiple supervised fully convolutional networks for the osteosarcoma segmentation of CT images. *Computer Methods and Programs in Biomedicine*.

[46] Ronneberger O., Fischer P., Brox T. U-net: convolutional networks for biomedical image segmentation.

[47] Lin T.-Y., Dollár P., Girshick R., He K., Hariharan B., Belongie S. Feature pyramid networks for object detection.

